# Association Rule Analysis of Influencing Factors of Literature Curriculum Interest Based on Data Mining

This article has been retracted.

**DOI:** 10.1155/2022/6866134

**Published:** 2022-05-21

**Authors:** Long Shi, Qingwei Zhu

**Affiliations:** College of Foreign Language, Pingdingshan University, Pingdingshan, Henan 467000, China

## Abstract

In recent years, the amount of educational data in colleges and universities has increased rapidly. Each university has set up multiple courses to recruit talents. Students cannot choose courses. The emergence of data mining technology and its application in college teaching and curriculum has been preferred particularly to streamline these activities. When analyzing the correlation of courses based on data mining technology, we usually use the correlation between the scores of various subjects to analyze the correlation between courses. Correlation among various courses that are offered at colleges or universities is reflected through many different aspects such as factors or metrics, which are affecting course interest, course content, course arrangement, etc. In this article, we have thoroughly analyzed various factors that are affecting students' interest in literature courses with the help of association rules of data mining technology. Through the collected original data, this article uses Apriori algorithm to screen the association rules affecting students' interest in literature courses and combines them with the current teaching situation to complete the rule analysis. The results of rule analysis show that the most relevant factors affecting students' interest in literature curriculum mainly include the space-time dimension of textbook selection and compilation, the processing method of selected reading, and the evaluation method. The reading content is effectively processed by using the counterpoint reading method, and the literature curriculum textbooks are compiled from the perspective of cross-cultural communication, to enhance students' interest in the literature curriculum.

## 1. Introduction

When studying the influencing factors of college literature curriculum interest, this article uses association rules for data analysis, which will generate a large number of rules and models. By analyzing the accurate rules in the data, that is, the literature classroom content that students are most interested in, this part adopts association rule analysis. The user's interest will be reduced due to the inconsistency between the rules and expectations, more noninteresting attributes in the rules, or more redundant rules. For this problem, attribute classification analysis should be adopted to clarify the front and rear items of association rules of data mining [1].

Data mining is a well-known concept, which is used for the extensive analysis and evaluation of data especially multivariate or univariate. However, data mining technology is a way of utilizing various algorithms, i.e., a benchmark which is available in the literature, to carry out the tedious task of dataset analysis. Additionally, it is used to find the high-value information in the data and use it in the interest correlation analysis of literature classroom, to find the data information consistent with the curriculum value in a large number of real data, realize the curriculum optimization, greatly improve the teaching quality, and cultivate more high-quality talents for the society [2].

The innovations in the research process of this article are (1) it uses data mining technology to analyze association rules and establish an association rule model in studying the influencing factors of interest in literature courses. By analyzing the factors affecting literature courses according to this process, we can get significantly related courses, further analyze and explain the relevant courses and obtain statistical significance factors, to analyze the correlation between courses and waiting courses [3]. (2) Relevant data have been refined through well-known fusion schemes, set minimum support and confidence thresholds to 0.2 and 0.83, respectively, and generate more than 500 rules. The results show the factors that affect the interest in literature courses are teaching methods, teaching materials, and assessment account for 30.8%, 27.8%, and 17.6%, respectively [4].

To resolve these issues, we have developed a unique way of effectively utilizing the Apriori algorithm to screen the association rules affecting students' interest in literature courses and combine them with the current teaching situation to complete the rule analysis. We have observed that the proposed scheme is very effective and convincing to resolve these issues, particularly with available resources and infrastructures. Various claims of this scheme have been verified through extensive simulations which are presented in the results section.

The remaining article is arranged according to the following agenda items. In Section 2, we have focused on the detailed description of the most related work especially those which are closely linked to the problem resolved in this article. In Section 3, a generalized and detailed description of the existing data mining algorithms and their usefulness have been presented along with various steps and flow diagrams where needed and applicable. In Section 4, association rules enabled data mining techniques have been presented and a detailed analysis is provided on how these techniques can resolve the issue under consideration in this article. Results of the simulations with various metrics have been presented in Section 5 which is followed by a comprehensive discussion or summary of the overall manuscript.

## 2. Related Work

Data mining technology was proposed in the 1980s and developed rapidly in the 1990s. In the science and technology review published by MIT, experts from Semenova pointed out that 3 of the 10 new technologies affecting human development in the next 5 years are related to data mining [5]. Many mature data mining algorithms have been developed abroad [6]. Mahmud has a high value in data mining. China has mainly carried out research on data mining algorithms and practical applications. Chen et al. obtained the dependence degree and dependence relationship between courses by analyzing students' course scores, to predict students' later course scores [7]. Sun et al. combine hierarchical association analysis and association rules to analyze students' graduation data and school performance, obtain the correlation between courses, important skills and core courses, establish a curriculum system based on a project-based curriculum teaching mode, and provide a reference basis for colleges and universities to improve courses [8]. Li et al. use the association rule algorithm to analyze the scores of various professional courses, which is used to judge the relationship between enterprise needs and courses, and provide teachers with the basis for improving teaching methods, to adjust the professional curriculum system [9]. Dou and Zhai use Apriori algorithm to study students' learning effect, better obtain the correlation between different courses, and early warning students' performance according to this relationship [10]. Predict the failing courses of the student union in advance, and focus on supervising the students' learning in the course. Wang et al. use data mining technology to establish an early warning model, use data statistics to complete low-level early warning, complete landslide early warning based on cluster analysis, find the relevance between different courses through association rule analysis, search the association rule base, predict the crisis in the process of students' learning, and improve the early warning effect [11]. Diao et al. use cluster analysis to record students' course selection information, study the commonalities of students when choosing courses of various majors, obtain the correlation between courses and grades based on score data, and formulate an ideal course selection group for various majors [12]. Xu et al. established the curriculum correlation analysis model based on a rough set and used the curriculum scores hidden in the curriculum correlation to guide students' course selection, to avoid students' blindness and uncertainty in course selection [13]. Sun et al. select the Apriori algorithm on SPSS association rules to analyze the relationship between the types of candidates, admission results, and regional grades, so that educators can quickly grasp the actual education level of a region and make educational decisions in combination with educational resources [14].

## 3. Data Mining Algorithm

### 3.1. Basic Concept and Process of Data Mining Algorithm

The definition of a data mining algorithm can be divided into broad sense and narrow sense. Generalized data mining refers to extracting the knowledge and decision content conducive to decision-makers in large-scale datasets. Data mining in a narrow sense is a process of mining knowledge of datasets stored in a fixed form. Machine learning and data mining are two different concepts. Data mining focuses on practical applications, whereas machine learning focuses on algorithms [15]. By using machine learning algorithms for data mining; using increasingly mature data mining patterns, rules, and mining tools; finding valuable laws according to the mining process; mastering the patterns and internal relations between different data; and using the data in practice to play a certain auxiliary role. On the whole, data mining consists of four stages, namely, the early data preparation stage, determination of mining mode stage, later development stage, and evaluation stage.  Figure 1 shows the flow chart of data mining.

1. **Data preparation:** data are the main part of data mining, so the preliminary preparation of data is very key. Most of the data come from different regions and different data types. These data are difficult in the process of data mining due to the lack of standardization. Therefore, before data mining, we should first master the data differences in various fields; learn industry knowledge, industry needs, and business processes; and determine the data mining objectives based on business needs.
2. **Data extraction:** data mining personnel extract the required data, delete all the data that is not valuable to the model, research the prepared integrated data, and clarify the value and scope of the data. Data miners should strictly follow the principle of data extraction in the stage of extracting data to ensure the realization of task objectives.
3. **Preprocessing data:** secondary processing of extracted data. This operation mode is to ensure that the data quality added to data mining meets the basic requirements, and the data consistency and integrity meet the requirements. For the source data from different systems, there are also differences in structure. Therefore, it is necessary to preprocess and clean the data to obtain unified data and ensure the high quality of the extracted data.
4. **Data mining:** by combining with industry data characteristics and system operation requirements, select the corresponding mining data and extract the valuable knowledge in the preprocessed data.
5. **Pattern evaluation:** deeply excavate interesting patterns and knowledge, and deliver them to experts for evaluation in a visual way. If some patterns fail to meet the task requirements, return to the above steps to further complete the operation until accurate patterns or knowledge are obtained.

### 3.2. Classification of Data Mining System

Data mining is a highly comprehensive discipline, which involves many fields and disciplines, such as statistics, database technology, information science, and machine learning, as shown in Figure 2. Accurately determine the type of data mining system to better mine the interests and hobbies of different users, and use the best mining tools to complete the data mining operation according to various classification standards. The main types of data mining systems are described as follows:

1. The database is divided into database types based on spatial data flow and relational data flow, including database types, database classification based on temporal data flow, etc.
2. Data mining-based knowledge type: according to data mining knowledge, it is divided into different types. The essence of its knowledge is a function, so it can be divided into data area, feature area, association analysis, clustering, classification and prediction, evolution analysis, and outlier analysis.
3. Application-based classification: different application areas have different specific data mining tasks, such as bioscience and telecommunications.

### 3.3. Clustering Analysis Algorithm

Clustering is a well-known concept in the research community which is used to divide various objects of different or similar properties into a defined number of classes. In physic, abstract objects or object classes with high similarity are clustering, and the collection of data objects is a cluster. The similarity between this object and objects in the same cluster is high, which is quite different from objects in other clusters [16]. It can be regarded as a cluster of data objects as a group, which is regarded as a form of compressed data. The automatic clustering algorithm can automatically identify each region in the object space, to obtain the internal relationship between the attribute set and the overall distribution pattern. At present, the application of cluster analysis in various fields, such as the use of cluster analysis in business activities, can help market decision-makers reasonably classify different customer types from the existing customer database and realize market segmentation. The clustering algorithm runs on the data matrix and dissimilarity matrix.

(1) Data matrix: *n* objects are represented by *P* variables, and the data structure is *n* × *p* matrix
  (1) $$\begin{array}{c} \left[\begin{array}{ccccc} X_{11} & ... & X_{1f} & ... & X_{1p}\\ ... & ... & ... & ... & ...\\ X_{i1} & ... & X_{if} & ... & X_{ip}\\ ... & ... & ... & ... & ...\\ X_{n1} & ... & X_{nf} & ... & X_{np} \end{array}\right]. \end{array}$$
(2) Dissimilarity matrix: saves the proximity of all paired *n* objects, and consists of the following *n* × *N* matrix representation:
  (2) $$\begin{array}{c} \left[\begin{array}{cccc} 0 & \; & \; & \;\\ d\left(2,1\right) & 0 & \; & \;\\ d\left(3,1\right) & d\left(3,2\right) & 0 & \;\\ ... & ... & ... & \;\\ d\left(n,1\right) & d\left(n,2\right) & ... & 0 \end{array}\right]. \end{array}$$

The *d*(*i*, *j*) represents the degree of difference between *i* and *j*, and *d*(*i*, *j*) is a non-negative value. The closer the value between the two objects is or the higher the similarity is, the closer the two values are to 0; the higher the value, the more difference between the two objects and the greater the degree of alienation. At the same time, *d*(*i*, *j*) = *d*(*j*, *i*), *d*(*i*, *i*) = 0.

When the variable type is a continuous scale value, the distance between two objects can be calculated based on the distance between each pair of objects. Nowadays, Manhattan distance and Euclidean distance are widely used.

The following is the definition of Euclidean distance:

(3) $$\begin{array}{c} d\left(i,j\right)=\sqrt{{\left(x_{i1}-x_{j1}\right)}^{2}+{\left(x_{i2}-x_{j2}\right)}^{2}+\cdots +{\left(x_{in}-x_{jn}\right)}^{2}}. \end{array}$$

These formulas *i* = (*X*_*i*1_, *X*_*i*2_,…, *X*_*in*_) and *j* = (*X*_*j*1_, *X*_*j*2_,…, *X*_*jn*_) are data objects with *n* dimensions. The Manhattan distance is defined by the following formula:

(4) $$\begin{array}{c} d\left(i,j\right)=\left|x_{i1}-x_{j1}\right|+\left|x_{i2}-x_{j2}\right|+\cdots +\left|x_{in}-x_{jn}\right|. \end{array}$$

## 4. Data Mining Based on Association Rules

Mining based on association rules is used to find the relationship between various items in the database. Using this rule to obtain students' interest in the literature classroom and relevant data, such as course content, course setting, course arrangement, and course innovation, all affect students' interest in the literature classroom [17]. Colleges and universities can use this rule to rearrange courses, set course contents, and further classify literature courses. However, this process needs a lot of data as support. We should extract students' relevant information about literature classrooms through data mining, to judge students' interest in the literature classroom and various factors affecting interest, and realize multilevel mining and analysis.

### 4.1. Association Rule Algorithm

The association rule algorithm is the most used in modern data mining. Imielinski, Agrawal, and Swami first proposed the association rule algorithm. The basic principle of the algorithm is to judge the influence on other phenomena by studying some phenomena. Generally, the rules required by load parameters are called strong association rules. In the 1990s, Agrawal scholars proposed the Apriori algorithm that is assumed as one of the best-suited schemes for the problems at hand. In this article, it is used especially breadth-first layer by layer iterative search method to obtain the frequent one item set. The polarity of the frequent two item sets is searched based on one item set, and the iterative analysis is carried out according to this order until the frequent item set cannot be found. The number of candidate sets generated by the Apriori algorithm is large, so it is necessary to prune them. And set ideal confidence and support as the screening conditions to improve and adjust the algorithm again, in which the support is the rule *A*⇒*B*, and the support is the frequency of frequent occurrence of two item sets a and B, that is, the frequency of occurrence of a and B at the same time in the intersection of U. Through the confidence degree, it is concluded that the transaction contains the probability of B, which can be expressed as *A*⇒*B*. Before carrying out the task, the task path should be replanned and the feasibility model should be constructed, and the quality of the model has a direct impact on the effect of data mining.

(5) $$\begin{array}{c} A\Rightarrow B. \end{array}$$

### 4.2. Build Model

The association rule mining-enabled model is completed in four steps, i.e., collecting data, mining data, interpreting data set, and applying data. During the practical application, the value and authenticity of data mining should be improved, and the results obtained are more objective. Generally, the original data collected is difficult to be processed directly by the algorithm, so it should be converted and adjusted according to the requirements of the algorithm. After that, the rules are used to explain and analyze it, and then combined with relevant experience and analysis results to analyze the interest in the literature curriculum [18]. This article constructs a model based on the characteristics of the literature curriculum and students' interest orientation, which is shown in Figure 3 [19].

## 5. Analysis of Association Rules of Influencing Factors of Literature Curriculum Interest Based on Data Mining

### 5.1. Data Mining and Rule Formation

When studying the influencing factors of interest in the literature courses, this article adopts the association rule analysis based on data mining. Based on the score data of college students' culture courses, the original data is preprocessed by denoising and discretization, and it is introduced into vs2012 software for association rule mining. The minimum support and minimum confidence thresholds are set to 0.2 and 0.83. After processing, more than 500 rules are generated. Screening the strong association rules according to the proportion obtained, the results show that among the factors affecting the curriculum of literary interest, teaching methods, teaching materials, and assessment accounted for 30.8%, 27.8%, and 17.6%, respectively, and other factors accounted for 23.8%.  Figure 4 shows the proportion of various factors affecting literature interest courses.

### 5.2. Rule Analysis

#### 5.2.1. Rule 1

Analysis rule 1 shows that most students are not interested in the traditional literature teaching mode. The proportion of selected students who express little interest in literature courses is 30.6%, and the confidence is 0.85. The students of multimedia teaching and textbook teaching mode are interested in the cultural connotation and interpretation of literature courses, accounting for 30.6%, and their confidence is 0.86. The teaching methods of literature history and selected literature courses are the least preferred, accounting for 35.8%, and the multimedia and textbook models are the most preferred, accounting for 41.5%. According to the results, the teaching mode, means, and processing selection methods directly affect students' interest in literature courses.  Table 1 shows the data mining results of rule 1.

Therefore, the most critical part of literature classroom teaching is selective reading, which accounts for more content in teaching materials. In addition, the use of modern online video technology can make classroom teaching more active. For example, in literary works, films, online video, e-chat, and other ways can be displayed in the form of images or sounds, so that students can intuitively experience the charm of literary works.

#### 5.2.2. Rule 2

Those who choose the first three results in the rule choose the last one, accounting for 20.3%, with a confidence of 0.87. If nonliterary works and literary works are fully integrated, it shows that students are more inclined to the ideological and cultural connotation curriculum, and the proportion of students who are a little interested in the cultural curriculum accounts for 88% [20]. The data mining results are shown in Table 2.

Based on the traditional teaching mode, the vividness and quality of teaching materials directly affect the teaching effect. After an in-depth analysis of the rules, the proportion of students who choose inclusive options is 51%, literature accounts for 42.9%, and nonliterature accounts for 12.6%. It can be seen that students' interest in the literature classroom is related to teaching materials. After analyzing the rules, the proportion of students choosing different cultural types can be seen in Figure 5.

#### 5.2.3. Rule 3

About 24.6% of the students surveyed were dissatisfied with the traditional teaching methods, expressed a little interest in the literature classroom opened by the school, were dissatisfied with the single teaching mode, but were interested in the selected reading content. About 53.7% of the students chose to be dissatisfied with the course paper, 36.4% of the students were dissatisfied with the literature class, and 2.4% of the students were dissatisfied with the examination method of the literature course.  Table 3 lists the data mining results of rule 3, and Figure 6 shows the proportion of students dissatisfied with the teaching method.

## 6. Conclusion

With the prevalence of national style, more and more people like literature, which has also attracted the attention of the field of education and all sectors of society. Under this environment, colleges and universities also began to pay attention to the literature classroom education, so that more people can learn deeper literature knowledge by setting up literature classrooms. However, during the study period, the learning effect is not ideal, and some students have low interest in the literature classroom, even truancy, and other phenomena. Aiming at this problem, this article uses the association rule analysis method based on data mining to study the influencing factors of interest in literature courses, deeply analyzes the association rule algorithm, establishes the association rule model based on data mining, obtains the data of students' interest in the literature classroom, and analyzes the educational methods that students like and dislike most. The results show that most students are dissatisfied with traditional teaching. According to the analysis of rule 1, only 30.6% of students are interested in literature courses and 41.5% are interested in the combination of multimedia teaching and textbook teaching. The least favorite teaching method is literature class and literature history, with a proportion of 35.8%. According to the analysis of rule 2, 51% of the students choose the type of inclusion items and 42.9% of the students choose the type of literature. Through the analysis of rule 3, it is concluded that 24.6% of the students are dissatisfied with the traditional teaching paradigm, 53.7% of the students are dissatisfied with the thesis course, 36.4% of the students are dissatisfied with the literature course, and 2.4% of the students are dissatisfied with the examination method of the literature course. This article uses Apriori algorithm analysis to find more factors that affect students' literature classroom and can find more hidden factors that affect students' performance, so that students' performance can be significantly improved.

## Figures and Tables

**Figure 1:** Data mining flow chart.

**Figure 2:** Disciplines involved in data mining.

**Figure 3:** Mining model of interest association rules in the literature curriculum.

**Figure 4:** Proportion of factors affecting literary interest curriculum.

**Figure 5:** Proportion of students choosing different cultural types.

**Figure 6:** Proportion of students dissatisfied with teaching methods.

**Table 1:** Data mining results of rule 1.

The serial number	In the preceding paragraph	Consequent	Support	Degree of confidence
Rule 1	The teaching mode that students are least interested in is the traditional knowledge mode, which is mainly taught by teachers in class and has little interaction with students. Pay more attention to the selected reading, you can roughly explain the content of the textbook, mainly on the ideological and cultural connotation of the selected reading analysis	Have some interest in the literature class	0.306	0.85
Referential rules	The teaching mode I am most interested in: multimedia + textbooks (such as videos, movies, and TV dramas): I pay more attention to the selected reading content, and it is better to explain the knowledge of textbooks roughly, focusing on the ideological and cultural connotation of the selected reading	Have some interest in the literature class	0.306	0.86

**Table 2:** Data mining results of rule 2.

The serial number	In the preceding paragraph	Consequent	Support	Degree of confidence
Rule 3	In the selected works, literature and nonliterature account for 50%, paying more attention to the content of the selected reading, which can be roughly explained in the works, focusing on the ideological and cultural connotation of the selected reading	Have some interest in the literature class	0.203	0.87
Referential rules	The textbook writers are mainly from China, and there are no literature works written by writers from other countries. The proportion of literature teaching works and personal selection works is half	Have some interest in the literature class	0.265	0.88

**Table 3:** Data mining results of rule 3.

The serial number	In the preceding paragraph	Consequent	Support	Degree of confidence
Rule 3	A little interested in literature class: the most dissatisfied is literature course papers, literature class, literature course assessment methods, traditional teaching mode, and selected reading: only interested in literary works of personal interest	Traditional single literature classroom teaching method	0.246	0.87

## Data Availability

The datasets used and analyzed during the current study are available from the corresponding author upon reasonable request.

## References

[1] Khedr A. M., Osamy W., Salim A., Abbas S. (2020). A novel association rule-based data mining approach for internet of things based wireless sensor networks. *IEEE Access*.

[2] Alsuwaiket M., Blasi A. H., Altarawneh K. (2020). Refining student marks based on enrolled modules’ assessment methods using data mining techniques. *Engineering, Technology & Applied Science Research*.

[3] Changpetch P. (2021). Multinomial logit model building via TreeNet and association rules analysis: an application via a thyroid dataset. *Symmetry*.

[4] Li J., Sacchi M. D. (2021). An l p -space matching pursuit algorithm and its application to robust seismic data denoising via time-domain radon transforms. *Geophysics*.

[5] Semenova N. S., Larichev A. V., Akopyan V. S. (2020). Swept source optical coherence tomography: a technology review. *Vestnik Oftalmologii*.

[6] Mahmood N., Hafeez Y., Iqbal K. (2021). Mining software repository for cleaning bugs using data mining technique. *Computers, Materials & Continua*.

[7] Chen M. S., Yang R., Tian H. G., Wang Z., Wang Y. (2021). Analysis of students’ higher Mathematics course results in Xijing University. *Modern Business Trade Industry*.

[8] Sun J., Zhang W., Ren Z. J., Wang D. L., Cui Y. (2017). Practice on OBE evaluation architecture for the achievement of graduation requirements based on the engineering education accreditation system. *Tsinghua Journal of Education*.

[9] Li J. L., Chu L. Q., Gui L., Hu B. (2018). Analysis and reflection on main course examination results of vocational nursing students from different sources. *China Continuing Medical Education*.

[10] Dou J., Zhai S. P. (2018). Research on early warning system of college student achievement based on improved apriori algorithm. *Modern Informationn Technology*.

[11] Wang D., D H., Wang Q. L. (2020). Research and application for early warning of landslides based on hierarchical clustering coupling weighting Markov chain model[J]. *Journal of China Coal Society*.

[12] Diao S., Chen L. W., Ma Y., Zhang T. (2019). Application of data envelopment analysis in individualized learning of health statistics[J]. *Chinese Journal of Health Statistics*.

[13] Xu W. Y., Wang Z. N., Wang P. X. (2017). Investigation and analysis on the influencing factors of finding satisfactory jobs for college students[J]. *Journal of Huaiyin Institute of Technology*.

[14] Sun F., Ren F. D., Shi S. Y., Tan Q. (2020). Application of association rule Apriori algorithms in analysis of the high school entrance examination score. *Journal of North China Institute of Aerospace Engineering*.

[15] Hernández J. F., Díaz Z., Segovia M. J., del Pozo E. (2020). Machine learning and statistical techniques. An application to the prediction of insolvency in Spanish non-life insurance companies[J]. *International Journal of Digital Accounting Research*.

[16] Ramkumar P., Kalamani P., Valarmathi C., Devi M. S. (2021). An effective analysis of data clustering using distance-based K- means algorithm[J]. *Journal of Physics: Conference Series*.

[17] Istiani I., Anam Z. (2021). Journal of literature, linguistics and culture studies integrating peace education in literature class. *Rainbow Journal of Literature Linguistics and Cultural Studies*.

[18] Kokhan R., Matsevko-Bekerska L., Lysanets Y. (2020). Conversation analysis tool as an effective means for teaching the university courses of English and world literature. *Arab World English Journal*.

[19] Yang M., Fan X., Xu H. R. (2020). Research on application of user interest model and Apriori algorithm in employment recommendation of college students. *Modern Electronics Technique*.

[20] Liu X. W. (2021). On approaches to integrating guilin anti-japanese war cultural resources into the ideological and political courses in Universities and Colleges. *Journal of Guilin Normal College*.

